The article "Effect of Zhujingqiaoyun Receptivity of Infertility with Kidney Deficiency Based on Ultrasonic Evaluation" was published in 2022. Journal: Evid Based Complement Alternat Med.

# Effect of Zhujingqiaoyun Receptivity of Infertility with Kidney Deficiency Based on Ultrasonic Evaluation

**DOI:** 10.1155/2022/3675689

**Published:** 2022-04-21

**Authors:** Xiaoli Mao, WeiMao, Ling Zhong, Zhun Qu, Huimin Chen, Qiaomin Wang, Jingjing He

**Affiliations:** ^1^Wuhan Hospital of Traditional Chinese Medicine, Wuhan, China; ^2^Department of Huawei Outpatients, Peking University Shenzhen Hospital, Shenzhen, China

## Abstract

**Objective:**

This study aims to explore the effect of the prescription for Zhujingqiaoyun receptivity in patients with infertility.

**Methods:**

This project is a prospective randomized controlled clinical study, including infertility diagnostic criteria and dialectical kidney deficiency patients. 60 cases were randomly divided into 2 groups: the control group, where medication complex packing estradiol tablets were given, and the treatment group, on the basis of the control group, which was given Zhujingqiaoyun receptivity plus or minus. Transvaginal ultrasound was used to observe the endometrial thickness, endometrial volume, endometrial blood supply, and other aspects of patients in the two groups to evaluate the endometrial receptivity before and after treatment, and to record the pregnancy rate and safety of patients in the two groups after three menstrual cycles.

**Results:**

There was no significant difference in age, course of disease, and endometrial thickness between the two groups (*P* > 0.05). Before and after treatment, the endometrial thickness of the two groups increased significantly, and the uterine artery blood flow pulsatility index (PI) and resistance index (RI) decreased significantly (*P* < 0.05). The endometrial volume in the control group was significantly lower than that in the treatment group, and the difference was statistically significant (*P* < 0.05). The endometrial FI and VFI in the control group were significantly lower than those in the treatment group, and the difference was statistically significant (*P* < 0.05). In the treatment group, 30 cases were treated for 3 months, and 11 of those were pregnant (36.7%). There were 30 cases in the control group, and 5 cases were pregnant (16.67%). Both groups had good safety. SPSS 22.0 statistical software was used for the chi-square test.

**Conclusion:**

Zhujingqiaoyun receptivity on endometrial receptivity can treat infertility patients with good efficacy, increasing endometrial thickness and reducing uterine artery blood flow index. It is worthy of clinical promotion to improve pregnancy rates.

## 1. Introduction

Couples who live together for one year without contraception and have a normal sex life and fail to conceive are called infertile. Infertility is one of the three major diseases affecting human life and health. At the same time, infertility is also a difficult disease that causes common concern all over the world. According to the relevant survey data, the incidence rate of infertility in China is 10% to 15%. One of the main reasons for female infertility is ovulation disorders. Ovulation-related infertility accounts for 25% to 30% of the causes of infertility [1]. The latter mainly depends on endometrial receptivity. Improving endometrial receptivity and increasing the implantation rate is the key to improve the pregnancy rate.

Endometrial receptivity means that the endometrium is in a state where the blastocyst can be positioned, adhered, and invaded, and the endometrial stroma changes at the same time, which leads to embryo implantation [2]. The embryo can be implanted smoothly, and excellent endometrial receptivity is essential. There are many clinical indicators to evaluate endometrial receptivity. Pinocytosis is a morphological indicator. Its acquisition is an invasive operation, and its clinical application is limited. Nowadays, three-dimensional color ultrasound is often used to monitor endometrial anatomy and physiological parameters to indirectly reflect endometrial receptivity [3]. Traditional Chinese medicine believes that the kidney is the main reproductive organ. For the treatment of infertile patients, Cang Fu Dao Tan decoction is added to strengthen the spleen and reduce phlegm. Phlegm wet removal can promote the development of follicles and improve the pregnancy rate [4, 5]. To improve the endometrial capacity, traditional Chinese medicine believes that tonifying the kidneys and promoting blood circulation is important [6]. Studies have found that the use of kidney-tonifying traditional Chinese medicine can thicken endometrial thickness and improve uterine arterial blood supply, thereby improving endometrial tolerance and increasing clinical pregnancy rate [7]. It is found that in traditional Chinese medicine, kidney deficiency and blood stasis are the main pathogenesis of low endometrial receptivity. Traditional Chinese medicine can improve endometrial receptivity and pregnancy rate by reducing blood flow resistance, increasing endometrial thickness, and improving endometrial type and endocrine hormone environment [6]. The theory of traditional Chinese medicine believes that the kidney is the main reproductive. The kidney is the origin of the congenital, and the spleen is the origin of the acquired, so the treatment is based on tonifying the kidney and strengthening the spleen, regulating Chong Ren, and has achieved good clinical effect. This study showed that the basic pathogenesis of the disease was based on deficiency, kidney deficiency, phlegm and blood stasis, so attention should be paid to the combination of promoting blood circulation and tonifying the kidney and spleen in treatment [8]. The formula in this test consists of tonifying the kidney and spleen, regulating qi, reducing phlegm and promoting blood circulation, taking dryness and dampness as the basic laws, as well as tonifying the kidney and promoting blood circulation. The whole party played kidney-tonifying spleen, resolving phlegm and promoting blood circulation [9].

In recent years, Chinese medicine has made some progress in the etiology, pathogenesis, treatment, curative effect observation, and mechanism of infertility. Dr. Shengyang Xu, a national-famous and old traditional Chinese medicine practitioner, summarized the previous experience and combined it with his own clinical experience for many years, putting forward that the disease is based on kidney deficiency, mixed with phlegm dampness or blood stasis. In the treatment, the method of tonifying the kidney, activating blood circulation, and resolving phlegm is adopted, which has significant curative effects in inducing ovulation, improving endometrial receptivity, and improving the pregnancy rate. Therefore, this study intends to explore the effect of the prescription for Zhujingqiaoyun receptivity in patients with infertility.

## 2. Methods

### 2.1. Participants

This study was verified by the Research and the Ethics Committee of Wuhan Hospital of Traditional Chinese Medicine, where the patients recognized the study procedure by signing the consent form and approval letter. This unit was facilitated with the staff having a specialized multidisciplinary team, comprising physiotherapy, dietetics, occupational therapy, medical and nursing.

By the principle of randomized control, 60 infertile women were divided into two groups: the treatment group and the control group, with 30 cases in each group.

The inclusion criteria were as follows: (1) meet the diagnostic and syndrome differentiation criteria of traditional Chinese medicine and Western medicine; (2) the reproductive ability of the spouse is normal; (3) the size and shape of uterus and ovary are normal after imaging and laparoscopy, and at least one fallopian tube is unobstructed after salpingography or hydrotherapy; (4) ovulation occurred in 3 natural ovulation cycles monitored by B-ultrasound; (5) no history of estrogen/progesterone uses within 3 months before admission; (6) there was no history of pelvic and uterine surgery within 6 months before admission; (7) sign informed consent; and (8) approved by the ethics committee.

The exclusion criteria were as follows: (1) a history of endocrine diseases; (2) endometritis and *tuberculosis*; (3) there are uterine malformations, endometriosis, and other diseases that cause abnormal uterine cavity morphology and lead to infertility; (3) received sex hormone treatment in recent 3 months; and (4) those who are allergic to drugs or allergic constitution.

### 2.2. Study Protocol

Control group: oral complex packing estradiol tablets were given from the 5th day of menstrual or withdrawal bleeding. 1 tablet, quaque die (qd), 21-day continuous treatment is a course of treatment. The drug is stopped for 1 week, regardless of menstrual cramps. The abovementioned steps were repeated for treatment for 3 consecutive courses.

Treatment group: on the basis of the control group, oral prescription for Zhujingqiaoyun receptivity (12 g *Rehmannia glutinosa*, 15 g *Cuscuta chinensis* Lam., 15 g *Morinda officinalis*, 15 g *Cistanche salsa*, 12 g *Cornus officinalis*, 15 g Lyciumbarbarum L., 15 g *Carapax Testudinis*, 10 g *Angelica sinensis*, 5 g *Rhizoma Chuanxiong*, 12 g *Paeoniae Radix* Alba, 15 g *Salvia miltiorrhiza* Bunge, 10 g *Rhizomacyperi*, and 12 g *Rhizoma Atractylodis* macrocephalae) was added. Decoction of traditional Chinese medicine in accordance with the requirements of “Management Regulations of Traditional Chinese Medicine Decoction Room in Medical Institutions” issued by the National Chinese Medicine (2009) No. 3, using drinking water that meets national health standards for decoction. Each dose of Chinese medicine was concentrated and filtered into 2 bags of liquid medicine, 200 ml/bag, divided into morning and evening. Starting from the fifth day of menstruation, one payment was made every day, and 21 days were taken as a course of treatment. The medication is stopped for 1 week. After menstrual cramps, the abovementioned steps were repeated for 3 consecutive courses of treatment. The medication was stopped in the case of pregnancy. Cold, greasy, and irritating foods were avoided during the medication.

### 2.3. Observation Index and Curative Effect Standard

After pregnancy determination treatment, blood/urine human chorionic gonadotropin (HCG) was detected. If it is (+), it indicates pregnancy. Then, the clinical pregnancy was diagnosed by transvaginal ultrasonography (35 days after ovulation) as an intrauterine gestational sac, fetal bud, or fetal heart. Pregnancy rate = number of clinical pregnancies/total number of cases × 100%.

Transvaginal three-dimensional color Doppler detection: (1) when the whole segment of the endometrium is displayed on the sagittal section of the uterus by transvaginal two-dimensional color Doppler, the thickness of the double-layer endometrium is measured at the place 10 mm away from the uterine fundus. After three consecutive measurements, the average value is calculated to observe the endometrial type and endometrial peristalsis. At the same time, after adding color on the sagittal section of the uterus, at the junction of myometrium and endometrium, the Doppler spectrum was taken out from the brightest part of the color blood flow of the low return vocal cord. The PI and RI were measured, and the average value was calculated after three consecutive measurements. (2) The 3D function key was enabled, the multiplane mode was applied, the volume angle to 120° was set, the sampling frame was adjusted to fully wrap the inner membrane, and the 3D volume data were obtained and stored after starting the volume scanning. The virtual organ computer-aided analysis (vol) software was used to draw the contour manually. The angle between each face of the extracted volume data was set to 30°. The intimal contour was drawn, 6 different sections were traced, and the three-dimensional volume of the intima was automatically obtained.

### 2.4. Statistical Analysis

SPSS 22.0 statistical software was used for data analysis. When the measurement data conform to the normality and homogeneity of variance, the mean ± standard deviation (*x* ± *s*) is used for statistical description. *P* < 0.05 was statistically significant, *P* < 0.01 was statistically significant.

## 3. Results

### 3.1. General Information Comparison

There was no significant difference in age, course of disease, and endometrial thickness between the two groups (*P* > 0.05) (Table 1).

### 3.2. Comparison of Efficacy Indexes between the Two Groups before and after Treatment

Before and after treatment, the endometrial thickness of the two groups increased significantly (Table 2 and Figure 1), and the uterine artery blood flow PI and RI decreased significantly (*P* < 0.05). The endometrial volume in the control group was significantly lower than that in the treatment group, and the difference was statistically significant (*P* < 0.05). The endometrial FI and VFI in the control group were significantly lower than those in the treatment group, and the difference was statistically significant (*P* < 0.05) (Table 3).

### 3.3. Comparison of Pregnancy Rate between Two Groups after Treatment

In the treatment group, 30 cases were treated for 3 months, and 11 of those were pregnant (36.7%). There were 30 cases in the control group, and 5 cases were pregnant (16.67%). It could be seen that the pregnancy rate of the experimental group was significantly higher than that of the control group, but the difference was not statistically significant by the chi-square (X^2^) test (*P* = 0.82) (*P* > 0.05).

### 3.4. Safety Observation

There was 1 patient in the treatment group who had mild diarrhea during medication, which did not affect normal work and life and was not treated with special treatment, but spontaneously relieved after two days. In the control group, 2 patients showed nausea symptoms, which did not affect their normal work and life, did not stop treatment, and then were relieved by themselves. No adverse reactions occurred in other patients. There were no abnormalities in blood and urine routine, electrocardiogram, liver and kidney function before and after treatment.

## 4. Discussion

Traditional Chinese medicine believes that the kidney stores the essence and governs reproduction and is connected to the uterus through the veins, which is the innate foundation and the root of gestation [10]. The essence of the kidney is filled, the qi and blood flow through the channels, and the endometrium is nourished, which is the material basis for the implantation of the fertilized egg and the continued pregnancy [11, 12]. Insufficient kidney essence, lack of source of essence and blood, inability to promote the circulation of qi and blood, endometrial and embryonic uterus cannot be nurtured, the uterus is unable to consolidate the fetal element, the material basis for gestation and growth is lacking, and the fetus loses its implantation soil, leading to infertility. Western medicine believes that after the fertilized egg is implanted into the endometrium, the growth of the endometrium must be synchronized with the fertilized egg to ensure the stability of embryo implantation [13]. This stability is called endometrial receptivity. Western medicine mainly improves the endometrial capacity by supplementing progesterone, estrogen, and using anticoagulant drugs, and strives to synchronize with follicular development, but the coordination is not good. Clomiphene citrate tablets have the effect of promoting ovulation and are currently commonly used drugs for the treatment of infertility, but they can inhibit the synthesis of estrogen, causing retardation of endometrial growth, a high ovulation rate, but a low pregnancy rate [14].

At present, the application of endometrial thickness to evaluate endometrial receptivity is still controversial. Some scholars believe that pregnancy rates decrease significantly when endometrial thickness is less than 7 mm. Dickey et al. [15] found that endometrial thickness in the pregnant group was significantly higher than that in the nonpregnant group, and they believed that endometrial thickness was an important factor in predicting pregnancy. However, Zollner et al. [16] believed that endometrial thickness had no statistical difference between pregnant and nonpregnant women and could not predict pregnancy. The endometrial thickness of the two groups after treatment was significantly different from that before treatment (*P* < 0.05). The therapeutic effect was better in the treatment group. It indicates that in the treatment of infertility patients, adding the treatment of Zhujingqiaoyun receptivity can increase the endometrial thickness.

Three-dimensional energy Doppler ultrasound can evaluate all blood vessels in the overall volume of an organ or tissue, which can accurately, intuitively, and truly reflect the blood perfusion in the area of interest. The parameters include VI, vascular index, which represents the ratio of color voxel value in the region of interest to the total voxel and represents the vascular density within the observed intimal volume, expressed as a percentage. The FI, or blood flow index, is interested in all color voxel intensity averages (i.e., the sum of the weighted color voxel divided by the total number of all the colors of the body element), which is all the average color value of blood flow or blood cell density. This prompts interest in the endovascular blood cell energy reflected by endovascular blood, the more the FI, the higher. VFI refers to the average color intensity of the total voxels in the area of interest; that is, the sum of all the color voxels divided by all the voxels. VFI reflects not only the vascular density of the tissue but also the blood cell density of the tissue [17]. The results of this study show that the endometrial volume in the control group was significantly lower than that in the treatment group, and the difference was statistically significant (*P* < 0.05). The endometrial FI and VFI in the control group were significantly lower than those in the treatment group, and the difference was statistically significant (*P* < 0.05).

In the treatment group, there were 30 patients, 11 of whom were pregnant after treatment, with a pregnancy rate of 36.67%. In the control group, there were 30 patients, 5 of whom were pregnant after treatment, and the pregnancy rate was 16.67%. The pregnancy rate in the treatment group was significantly higher than that in the control group, but the difference was not statistically significant (*P* > 0.05), which may be related to the small sample size and short treatment time.

## 5. Conclusion

According to the results of the trial, Zhujingqiaoyun receptivity on endometrial receptivity can increase the endometrial thickness and improve the endometrial type of infertility patients on ovulation day, reduce the uterine artery blood flow resistance, and other endometrial receptivity indicators. Therefore, Zhujingqiaoyun receptivity can treat infertility patients with good efficacy, increasing endometrial thickness, and reducing uterine artery blood flow index. It is worthy of clinical promotion to improve pregnancy rates.

## Figures and Tables

**Figure 1:** (a, b) After three-dimensional power Doppler imaging, the endometrial volume of the two groups was measured by voice software. (c) (d) After three-dimensional power Doppler imaging, the blood flow histogram function was used to obtain the endometrial VL, FI, and VFI of the two groups.

**Table 1:** General information comparison.

Group	N	Age	Course of disease	Endometrial thickness (mm)
Control group	30	28.62 ± 3.72	4.65 ± 1.06	7.35 ± 0.98
Treatment group	30	28.43 ± 3.27	4.72 ± 1.24	7.31 ± 0.84

**Table 2:** Comparison of three-dimensional ultrasonic parameters between two groups after treatment.

Group	N	Endometrial volume	VI%	FI	VFI
Control group	30	3.76 ± 0.78	4.65 ± 1.06	23.07 ± 2.58	1.12 ± 0.38
Treatment group	30	5.23 ± 0.84^*∗*^	4.72 ± 1.24	24.36 ± 2.18	1.26 ± 0.29

*Note.P* < 0.05^*∗*^.

**Table 3:** Comparison of efficacy indexes between the two groups before and after treatment.

Group	N	Time	Endometrial thickness (mm)	PI	RI
Control group	30	Before treatment	7.35 ± 0.98	2.53 ± 0.72	0.92 ± 0.12
		After treatment	7.87 ± 0.86	2.49 ± 0.68	0.86 ± 0.08

Treatment group	30	Before treatment	7.31 ± 0.84	2.56 ± 0.80	0.90 ± 0.10
		After treatment	8.34 ± 0.91^*∗*^	2.31 ± 0.55	0.81 ± 0.07

*Note.P* < 0.05^*∗*^.

## Data Availability

The data used to support this study are available from the corresponding author upon request.
